# Loss of a Conserved tRNA Anticodon Modification Perturbs Plant Immunity

This article has been retracted.

**DOI:** 10.1371/journal.pgen.1005586

**Published:** 2015-10-22

**Authors:** Vicente Ramírez, Beatriz Gonzalez, Ana López, María José Castelló, María José Gil, Bo Zheng, Peng Chen, Pablo Vera

**Affiliations:** 1 Instituto de Biología Molecular y Celular de Plantas, Universidad Politécnica de Valencia-C.S.I.C, Ciudad Politécnica de la Innovación, Valencia, Spain; 2 College of Horticulture and Forestry Sciences, Huazhong Agricultural University, Wuhan, China; 3 National Key Laboratory of Crop Genetic Improvement and National Centre of Plant Gene Research, HuaZhong Agricultural University, Wuhan, China; The University of North Carolina at Chapel Hill, UNITED STATES

## Abstract

tRNA is the most highly modified class of RNA species, and modifications are found in tRNAs from all organisms that have been examined. Despite their vastly different chemical structures and their presence in different tRNAs, occurring in different locations in tRNA, the biosynthetic pathways of the majority of tRNA modifications include a methylation step(s). Recent discoveries have revealed unprecedented complexity in the modification patterns of tRNA, their regulation and function, suggesting that each modified nucleoside in tRNA may have its own specific function. However, in plants, our knowledge on the role of individual tRNA modifications and how they are regulated is very limited. In a genetic screen designed to identify factors regulating disease resistance and activation of defenses in Arabidopsis, we identified *SUPPRESSOR OF CSB3 9* (*SCS9*). Our results reveal *SCS9* encodes a tRNA methyltransferase that mediates the 2´-*O*-ribose methylation of selected tRNA species in the anticodon loop. These SCS9-mediated tRNA modifications enhance during the course of infection with the bacterial pathogen *Pseudomonas syringae* DC3000, and lack of such tRNA modification, as observed in *scs9* mutants, severely compromise plant immunity against the same pathogen without affecting the salicylic acid (SA) signaling pathway which regulates plant immune responses. Our results support a model that gives importance to the control of certain tRNA modifications for mounting an effective immune response in Arabidopsis, and therefore expands the repertoire of molecular components essential for an efficient disease resistance response.

## Author Summary

Numerous studies revealed the existence of nearly 110 ribonucleoside structures incorporated as post-transcriptional modifications in tRNA, with 25–30 modifications present in any one organism. Emerging evidence points to the critical role of tRNA modifications in various cellular responses to stimuli, including transcription of stress response genes and control of cell viability and growth. The primary function of tRNA modifications, and in particular tRNA methylations, are linked to different steps in protein synthesis including stabilization of tRNA structures, reinforcement of the codon-anticodon interaction, regulation of wobble base pairing, and prevention of frameshift errors. Furthermore, tRNA methylations are involved in the RNA quality control system and regulation of tRNA localization in the cell, all of which affect translation rate, but modifications in the anti-codon, which exhibit important roles in decoding mRNA are particularly important. We identified that the *SCS9* gene from Arabidopsis encodes a tRNA 2´-O-ribose methyltransferase homologous to the TRM7 methyltransferase from yeast. We identify that SCS9 is crucial for the 2´-*O*-ribose methylation of nucleotides 32 and 34 of the tRNAs anticodon loop of certain tRNA molecules. We show that SCS9 is required for effectiveness of plant immunity and suggest the importance of precise tRNA modifications in this process.

## Introduction

Transfer RNA (tRNA) is a noncoding RNA responsible for the accurate addition of an amino acid to the 3´ end of a translating protein, and therefore functions as an adapter molecule responsible for decoding mRNA into the corresponding peptide sequence. tRNA molecules are 75–78 nucleotides long with a distinct three-dimensional L-shape, often represented in two dimensions as a cloverleaf to display each of the four stem-loop arms (acceptor arm, variable D arm, anticodon arm, and variable/TΨC arm) generated by internal base pairing. An additional distinguishing feature of tRNA is that among the 107 post-transcriptional modifications found in RNA, 92 of these modified nucleosides are present on tRNA molecules [1]. Interestingly, the biosynthetic pathway of the majority of tRNA modifications include at least a methylation step, and the number of modified bases varies among individual tRNA types, and among different prokaryotes and eukaryotes species. Modifications vary from a single methylation on the ribose to complicated side chains modifications in different positions on the purine/pyrimidine ring [1–3]. Comprehensive information on structures and positions of these modifications in tRNA molecules, tRNA biosynthetic pathways, and responsible enzymes are deposited in different RNA modification databases (e.g., http:modomics.genesilico.pl/). Nucleoside tRNA modifications remain extensively studied in bacteria and yeast, and data has most recently been reported in humans. Most biochemical pathways and genes encoding modification enzymes were identified from these studies. The fact that post-transcriptional modifications are highly conserved, based on the variety of organisms reported, underscores their importance. In bacteria and *S*. *cerevisiae*, the relationship between type and quantity of modified nucleosides in tRNA molecules and metabolism has been suggested as a regulatory device acting as biological sensors, continually adjusting based on growth conditions [3,4,5]. However, little is documented on tRNA-modified nucleosides in plants, and research in genetic and biochemical regulation is still in its infancy. However, a recent study performed in Arabidopsis and hybrid aspen (*Populus tremula x tremuloides*) identified 21 modified nucleosides in tRNAs in both species [6]. In addition, very few plant tRNA sequences are available to identify modified nucleosides on different positions of individual tRNA species, and very few plant tRNA modifying enzymes have been purified or identified [6–9].

*S*. *cerevisiae* cytoplasmic tRNAs have on average 12.6 modifications per tRNA, with 2.6 modifications occurring within the anticodon loop (N_32_-N_38_), and the remaining 10 modifications occurring in the main body of the tRNA, remote from the anticodon loop [10]. This ratio and distribution of modifications seem to be conserved in mammalian tRNA. Modifications in the main body of the tRNA appear crucial for stability of the molecule, with the absence of certain body modifications eliciting a quality control pathway which results in the degradation of specific tRNAs at different stages of biosynthesis [11]. Instead, many tRNA modifications that occur in the anti-codon loop play several crucial roles in translation [4,12]. Some of these modifications exhibit a role in ensuring charging fidelity, while others affect decoding efficiency and/or accuracy, presumably by altering codon:anticodon interactions in the ribosome. Several other modifications in and near the anticodon loop also affect reading-frame maintenance. Modified nucleoside deficiencies can therefore lead to reduced translation efficiency and increased errors, which will affect gene expression regulation and cell metabolism. In the majority of cases, however, it is not clear exactly which tRNA are affected by a lack of specific anticodon loop modifications, how the absence of modification explains the observed phenotype, and exactly how the alteration influences individual translation steps. One such important modification is the concurrent 2´-*O*-methylation of N32 and N34. The latter occupies the anticodon wobble nucleotide, which forms Nm32 and Nm34 in the anticodon loop, and is critical for tRNA function, but remains largely unexplored. In yeast, 2´-*O*-methylation occurs on C32 and N34 of tRNA^Phe^, tRNA^Leu^ and tRNA^Trp^ and requires Trm7 methyltransferase; and *trm7* mutant strains showing growth reduction, presumably due to translation defects [13]. Trm7 and the associated modifications are of particular interest for two additional reasons. First, 2´-*O*-methylation of the anticodon loop is highly conserved in eukaryotes. Thus, all five sequenced eukaryotic tRNA^Trp^ species have Cm32 and Cm34, and all 17 sequenced eukaryotic tRNA^Phe^ genes have Cm32, 16 of which also possess Gm34 [10]. Second, Trm7 and its modifications are associated with human disorders. Mutations in the putative TRM7 homolog FTSJ1, have been strongly associated with non-syndromic X-linked mental retardation in multiple studies [14], and tRNA^Phe^ from neuroblastoma cells and Ehrlich ascites tumors has a substantial portion of its tRNA^Phe^ lacking Cm32 and Gm34 [15]. Despite growth defects in yeast *trm7*-Δ mutants, widespread conservation of 2´-*O*-methylation of the anticodon loop, and the likely importance of FTSJ-mediated modifications in humans, no evidence exists to date supporting the importance of this tRNA modification type in plants, and the consequences of a failure in its control by TRM7 homologous genes. Moreover, while nucleoside tRNA modifications are commonly reported in bacteria and yeast, where most of the biochemical pathways and genes encoding modification enzymes have been identified, the study of tRNA modified nucleosides in plants has rarely been documented. The presence of modified nucleosides is well accepted but information on modifying enzymes in plants is scant.

The present study provides insights into the functional implications that some specific tRNA modifications at the anticodon loop had on the activation of an efficient disease resistance response in Arabidopsis towards the bacterial pathogen *Pseudomonas syringae* DC3000, the causal agent of bacterial speck disease. During a search for genetic suppressors in Arabidopsis for the enhanced disease resistance *csb3* mutant [16], we identified the *SCS9* gene (standing for suppressor of *cs* *b3*) which encodes a functional homologue of the methyltransferase Trm7 from yeast. Our results provide evidence that SCS9 is crucial to maintain intact plant immunity towards the bacterial pathogen *P*.*s*. DC3000, with loss-of-function alleles abrogating plant immunity towards this pathogen. We employed genetic, molecular, and physiological analyses, and concluded it is vital to maintain 2´-*O*-methylation of the tRNA anticodon loop molecules intact to ensure plant immunity against *P*.*s*. DC3000. Therefore, our results uncover a new critical component required for disease resistance in Arabidopsis.

## Results

### *scs9* identification

Arabidopsis enhanced disease resistant *csb3* mutant was isolated during a search for negative disease resistance regulators [16]. Enhanced disease resistance to *P*.*s*. DC3000 occurred in *csb3* plants with increased accumulation of salicylic acid (SA) and constitutive expression of pathogenesis-related (*PR*) genes. Moreover, epistasis analysis with different genes involved in the SA signal transduction pathway revealed *csb3* plants required intact SA synthesis and its recognition through the NPR1 receptor [16].

We conducted a search for *csb3* suppressors in a screen for mutants to further our understanding of plant immunity. Hence, homozygous *csb3* seeds were re-mutagenized with ethyl methanesulfonate (EMS), and approximately 20000 M2 seeds were grown, and screened to identify individuals that no longer exhibited enhanced resistance to *P*.*s*. DC3000 attributable to the *csb3* mutation. This screen rendered the isolation of the recessive *scs9* (standing for suppressors of *cs* *b3*) mutant (Fig 1). *csb3 scs9* plants lost the distinguishable morphological and growth arrest phenotype of *csb3* plants (Fig 1A). Also, the pathogen-responsive marker *pP69C*::*GUS* gene [17], constitutively expressed in the single *csb3* mutant [16], was abrogated in the double *csb3 scs9* mutant (Fig 1B). Moreover, comparative observations of *P*.*s*. DC3000 growth rates in Col-0, *csb3*, and *csb3 scs9* infected leaves showed the *scs9* mutation blocks the characteristic enhanced resistance to *P*.*s*. DC3000 due to the *csb3* mutation (Fig 1C). Notably, *csb3 scs9* plants were far more susceptible to *P*.*s*. DC3000 than Col-0 plants, evidenced by a 100-fold increase in bacterial growth compared to *csb3* plants. Enhanced susceptibility of *csb3 scs9* plants to *P*.*s*. DC3000 was of a similar magnitude, if not higher, than that observed in *npr1* plants (Fig 1C). Furthermore, genetic analyses indicated the *scs9* mutation was extragenic to *csb3*, and when segregated from the *csb3* mutant background by backcrossing to Col-0 plants, the compromised immune response conferred by the *scs9* mutation alone was maintained in the absence of the *csb3* mutation (Fig 1C). The enhanced bacterial growth in the single *scs9* mutant was accompanied by distinguishable symptoms of induced chlorosis, presumably due to high levels of bacterial growth reached in the mutant (Fig 1D). In summary, these results indicate SCS9 represents an important locus regulating plant immunity to *P*.*s*. DC3000 in Arabidopsis.

**Fig 1:** Characterization of scs9 plants. (**A**) Comparison of Col-0, *csb3* and *csb3 scs9* plants at four weeks after sowing. Note the stunted phenotype of the single *csb3* mutant and the growth recovery conferred by the *scs9* mutation in the double *csb3 scs9* mutant. (**B**) Comparative histochemical analysis of GUS activity in rosette leaves from a parental wild-type Col-0 plant carrying the *pP69C*:*GUS* transgene, which shows no constitutive expression of the transgene (left), from *csb3* plants showing the constitutive activation of the transgene (center), and the reversion of this molecular phenotype in the double *csb3 sc*s*9* mutant plant (right). (**C**) Growth rates of virulent *P*.*s* DC3000 in Col-0, *npr1-1*, *csb3*, *csb3 scs9*, and *scs9* plants. Bacterial growth was measured at zero (white bars), three (grey bars), and five (black bars) days after inoculation. Error bars represent standard deviation (n = 12). Asterisks indicate statistical differences to Col-0 (P<0.05) using a Student’s t-test. (**D**) Representatives of *P*.*s*. DC3000 inoculated Col-0 and *scs9* plants, where the *scs9* mutant exhibits a distinguishable enhancement of chlorosis due to bacterial growth.

In summary, these results indicate *SCS9* represents an important locus regulating plant immunity to *P*.*s*. DC3000 in Arabidopsis.

### *scs9* plants retain intact components of innate and SA-mediated immunity

The enhanced disease susceptibility of *scs9* plants might result from a lack of pathogen recognition or defects at any step downstream in the signaling pathway leading to activation of plant immune responses. Insights into the level *scs9* might be operating were gained by studying major hallmarks of plant immune responses in search of defects that might explain the compromised mutant immunity. We first tested whether *scs9* plants might be affected in early recognition of pathogen-associated molecular patterns (PAMPs) by measuring PAMP-mediated deposition of the β-1,3-glucan cell wall polymer callose. The degree of callose deposition induction in PAMP-treated leaves was monitored after staining with aniline blue, examined by UV fluorescence microscopy (Fig 2A), and quantified by counting yellow pixels on digital images (Fig 2B). The response to the bacterial flagellar peptide elicitor flg22, or to chitosan, which are unrelated PAMPs that induce callose deposition in Arabidopsis, was similar in *scs9* and Col-0 seedlings (Fig 2A and 2B). *MYB51* gene expression [18] and mitogen-activated protein kinase (MAPK) activation [19,20] constitute additional hallmarks for early PAMP-mediated immune signaling. Induction of *MYB51* transcript accumulation, measured by RT-qPCR at 5, 10 and 60 min upon flg22 application, revealed no differences between Col-0 and *scs9* plants (Fig 2C). Early elicitation of MPK activation following flg22 application was visualized by employing an antibody that recognized the phosphorylated residues within the MAPK activation loop. Western blot analysis of protein extracts derived from Col-0 and *scs9* plants revealed positive immunoreactive signals in the two polypeptides corresponding to MPK6 and MPK3 (Fig 2D). Marked transient activation of both kinases occurred after flg22 application; activation was maximal at 5–10 min and then declined at 30 min, remaining only partially active at 120 min after treatment. Results revealed no differences between Col-0 and *scs9* plants with respect to the pattern of MAPK activation (Fig 2D). All these observations therefore indicated that the activation of early stage of basal immunity was not affected in the *scs9* mutant.

**Fig 2:** Characterization of the *scs9* mutant. (**A**) Callose deposition in Col-0 and *scs9* cotyledons following application of flg22 and Chitosan. Aniline blue staining and epifluorescence microscopy was applied to visualize callose accumulation. (**B**) Callose deposition was calculated as arbitrary units by quantifying the number of yellows pixels per million on digital micrographs of flg22- or chitosan-treated leaves at 24 h. Bars represent mean ± SD, n = 15 independent replicates. (**C**) Time-course RT-qPCR analysis showing *MYB51* gene expression in Col-0 and *scs9* plants after application of flg22. Data represent mean ± SD; n = 3 replicates. (**D**) Western blot with anti-pTEpY antibodies of crude protein extracts derived from Col-0 and *scs9* plants at 0, 5, 10, 30, 60, and 120 min after treatment with flg22. Below is shown a Western blot with an anti-AtMAPK6 antibody revealing that MPK6 protein accumulated to similar levels in all the samples. Equal protein loading was verified by staining of the nitrocellulose filter with Ponceau-S dye. The experiments were repeated three times with similar results. (**E**) Western blot with anti-pTEpY antibodies of crude protein extracts derived from Col-0, *scs9* and *npr1-1* plants at 0, 24, and 48 h.p.i with *P*.*s*. DC3000. Equal protein loading was verified by staining of the nitrocellulose filter with Ponceau-S dye. The experiments were repeated three times with similar results. (**F**) Free SA and conjugated SAG accumulation in Col-0 and *scs9* mutant at 0, 24, and 48 h.p.i with *P*.*s*. DC3000. Data represent the mean ± SD; n = 3 replicates. (**G**) Time-course RT-qPCR analysis showing *PR-1*, *PR-2*, *PR-4*, *PR-5*, *SBT3*.*3*, *and SID2* gene expression in Col-0 and *scs9* plants after infection with *P*.*s*. DC3000. Data represent mean ± SD; n = 3 replicates. (**H-I**) Western blots with anti-PR-1 antibody. **H**, inhibition of PR-1 protein accumulation in *npr1*, compared to Col-0 or in *scs9* mutant plants following inoculation with *P*.*s*. DC3000. **I**, induced accumulation of PR-1 protein following application of SA (50 μM) in Col-0 and *scs9* plants. Experiments were repeated three times with similar results.

We next sought to demonstrate if in a plant-pathogen interaction, like that following *P*.*s*. DC3000 inoculation, *scs9* plants might be defective in eliciting MPK activation. Western blot analysis of protein extracts derived from Col-0, *scs9*, and *npr1* plants, the latter used as a control of a mutant also compromised immunity, revealed positive immunoreactive signals in the two polypeptides corresponding to MPK6 and MPK3, which were visible at 24–48 hours post inoculation (h.p.i.) with *P*.*s*. DC3000 (Fig 2E). Results showed no notable differences among the three genotypes, suggesting *scs9* defects, as in *npr1*, were positioned downstream of MPK activation following pathogen perception.

Compromised synthesis or perception of salicylic acid (SA) is on the basis explaining the compromised immunity observed in different mutants (i.e. *sid2* or *npr1*, respectively) [21,22]. Consequently, we considered if *scs9* plants might carry defects in SA biosynthesis and/or its accumulation. Therefore, we conducted measurements to determine whether endogenous SA levels were affected in *scs9* plants. Free SA and conjugated salicylate glucoside (SAG) concentrations were comparatively examined in leaf tissues from *scs9* and Col-0 plants following *P*.*s*. DC3000 inoculation (Fig 2F). In *scs9* plants, basal and induced amounts of free SA equaled the levels observed in Col-0 plants. SAG content was consistent with SA (Fig 2F). This finding suggested that the increased pathogen susceptibility observed in *scs9* plants was not due to defects in SA biosynthesis.

We subsequently examined whether SA perception was defective in *scs9*, as detected in the *npr1* mutant, where compromised immunity was accompanied by the absence of induced SA-responsive gene expression [22]. Therefore, induced expression of several genes diagnostic of SA-mediated disease resistance was examined by RT-qPCR in *scs9* and Col-0 plants following inoculation with *P*.*s*. DC3000. SA-responsive *PR-1*, *PR-2*, *PR-4*, *PR-5*, and *SID2* gene expression profiles, or even the recently described *SBT3*.*3* gene, which is pivotal in plant immunity [23], showed no differences in *scs9* plants when compared with Col-0 at 0, 24, and 48 h.p.i. with *P*.*s*. DC3000 (Fig 2G). This indicated transcriptional reprogramming occurred in *scs9* plants following pathogen perception. This conclusion was further supported by Western blot analysis showing that induced accumulation of PR-1 protein after bacterial infection was similar in *scs9* and Col-0 plants at 24 h.p.i.; both genotypes showing higher accumulation of the protein at 48 and 72 h.p.i. with only a marginal difference in PR-1 protein accumulation observed in the mutant (Fig 2H and S1 Table). As expected, PR-1 accumulation was nearly absent in *npr1* plants, here used as a control (Fig 2H and S1 Table). These results revealed differences between *scs9* and *npr1* mutants, and suggested the mutations are not allelic. Moreover, notable accumulation of PR-1 protein in response to exogenous SA application was observed in *scs9* and Col-0 (Fig 2I); only a very slight reduction in PR-1 accumulation could be observed in *scs9* plants at 24 h after SA application (S1 Table) further corroborating that *scs9* plants show no severe defects in SA perception.

### *SCS9* is At5g01230 and encodes a 2´-*O*-ribose tRNA methyltransferase

The *scs9* position was mapped by outcrossing *scs9* to Landsberg *erecta* (L*er*) plants, and F2 plants were scored for co-segregation of enhanced susceptibility to *P*.*s*. DC3000 using simple sequence length polymorphisms (SSLPs). Thirty-five plants selected from a L*er* x *scs9* F_2_ population were analyzed and *scs9* was mapped to chromosome 5, in close proximity to the top telomeric region, and linked to marker SGCSNP13418. We next collected 80 F2 individuals with the *scs9* phenotype, isolated individual genomes, which were bulked and deep-sequenced using the Illumina GAIIx platform. The resulting data were analyzed using a bioinformatic pipeline devised by Austin *et al*. [24] to identify a genomic region where putative mutations of interest resided. Between the identified mapping intervals, we identified one nucleotide substitution corresponding to a G-for-A transition, as expected for a mutation caused by EMS mutagenesis. This resulted in a Ser-for-Asn substitution at position 194 of the protein encoded by the gene At5g01230 (Fig 3A). Therefore, *SCS9* should correspond to At5g01230.

**Fig 3:** *scs9* is a mutant allele of At5g01230. (**A**) *SCS9* corresponds to At5g01230. The G nucleotide residue mutated to an A nucleotide in the *scs9* allele is indicated in bold letters. The deduced amino acid sequences are indicated above each nucleotide sequence, and the deduced amino acid change (S194 to N194) is shown in bold. (**B**) Intron-exon arrangement in At5g01230. Exons are shown as boxes. The distances are only approximate. Position of a T-DNA insertion in the third intron (indicated by a black box) and localization of the EMS-induced mutation in the 9th exon, rendering *scs9-2* and *scs9-1* mutant alleles, are indicated. (**C**) RT-qPCR analysis of the *SCS9* transcript accumulation levels in mock- and *P*.*s*. DC3000-inoculated Col-0, *scs9-1*, and *scs9-2* plants at 3 d.p.i. Data represent the mean ± SD; n = 3 replicates. (**D**) Comparative growth of *P*.*s*. DC3000 in Col-0, *scs9-1*, *scs9-2*, and *npr1* plants 3 d.p.i. Error bars represent SD (n = 12). Below are representatives of inoculated leaves of the indicated genotypes. (**E**) *SCS9* overexpression complements the *scs9-1* mutant and bacterial growth titers reach Col-0 levels. Plants of the indicated genotype were inoculated with *P*.*s*. DC3000. Bacterial growth was measured zero (white bars), three (grey bars), and five (black bars) d.p.i. Error bars represent SD (n = 12). Asterisks indicate statistical differences compared with Col-0 (P<0.05) analyzed using a Student’s t-test.

We complemented the results of our cloning strategy by searching for existing *SCS9* mutant alleles in T-DNA insertion mutant collections. One insertion mutant allele was detected, named here as *scs9-2*, which interrupted the third intron of the At5g01230 transcribed region (Fig 3B). RT-qPCR analyses of *SCS9* transcript levels in *scs9-2* plants, compared to *scs9-1* or Col-0 plants, revealed the absence of transcript accumulation in the former mutant (Fig 3C). The experiment also revealed the *SCS9* gene was expressed in moderate levels in Col-0 and *scs9-1*; and expression did not change following plant inoculation with *P*.*s*. DC3000 (Fig 3C).

A comparison of disease resistance response to *P*.*s*. DC3000 between *scs9-1* and *scs9-2* plants showed both mutants were equally affected, indicating notable increased susceptibility. The heightened susceptibility was of a magnitude similar to that shown in *npr1* plants (Fig 3D).

Finally, to confirm At5g01230 corresponds with the *SCS9* gene, *Agrobacterium*-mediated plant transformation was used to introduce into *scs9-1* (*scs9OEXSCS9* plants) and Col-0 (*wtOEXSCS9* plants) a cDNA corresponding to At5g01230, fused in frame to GFP, and under control of the constitutive 35S CaMV promoter. Several transgenic lines were generated with the *35S*::*SCS9* construct and some were studied in detail. All transgenic lines generated lost the characteristic enhanced disease susceptibility to *P*.*s*. DC3000 attributable to the *scs9-1* mutation. Fig 3E compares bacterial growth for the following: i) a transformed line in the *scs9-1* genetic background (i.e., line 4.4); ii) transgenic line in the Col-0 background (i.e., line 7.4); and iii) both with respect to non-transformed *scs9-1* and Col-0 plants. *SCS9* expression restored enhanced disease susceptibility in *scs9-1* plants to Col-0 levels further supporting the conclusion that At5g01230 is *SCS9*.

An *in silico* genome search for homologous amino acid sequences revealed the highest similarity of SCS9 was to bacterial FtsJ/RrmJ [25], yeast Trm7p [13], and human FTSJ1 [26] proteins, all encoding 2´-*O*-ribose tRNA methyltransferases (MTases). S1 Fig shows the key conserved elements of the predicted AdoMet- and ribose-binding sites of these four tRNA methyltransferases, including the predicted catalytic tetrad of two basic and two acidic side chains (K28, D126, K166, and E201; each marked with a red triangle) [27], which is a conserved feature in many 2´-*O*-ribose methyltransferases exhibiting the common `MTase fold´ [9,28]. Arabidopsis SCS9 and the orthologous MTases from bacteria, yeast, and humans exhibited striking conservation to the predicted active site and its neighborhood, suggesting similarity to their target RNA.

Pintard *et al*. [13] proposed a tRNA substrate interaction model, and predicted the yeast Trm7 protein solvent-exposed side chain of S197 and R194 residues, equivalent to S199 and R196 in the Arabidopsis SCS9 protein, interacts specifically with the phosphate group of the methylated nucleotide. The *scs9-1* mutation is located where the conserved S194 is substituted by N194, and lies very proximal to the mentioned residues, and the catalytically important E201 tetrad residue. Therefore, it is very likely the *scs9-1* loss-of-function might be due to a lack of enzymatic activity, which would reveal the importance of the S194 residue for 2´-*O*-tRNA methyltransferases.

### SCS9 complements *trm7*Δ mutant cells in yeast

Similarity between Arabidopsis SCS9 and the *bona fide S*. *cerevisiae* Trm7p tRNA MTase amino acid sequences led us to investigate whether SCS9 might functionally mimic Trm7p. The deleted *S*. *cerevisiae trm7*Δ strain phenotype is characterized by slow growth compared with the wild-type strain [13]. Therefore, to examine whether the *SCS9* gene provided the functions of the fission yeast *TRM7* gene, we attempted complementation of a *trm7*Δ mutant strain. Unlike the vector alone (Fig 4A), the yeast/*E*.*coli* shuttle vector carrying the *SCS9* cDNA complemented the *trm7*Δ mutant slow growth phenotype (Fig 4A). We therefore concluded the *SCS9* gene is the Arabidopsis functional homolog of the *TRM7* gene.

**Fig 4:** Complementation of the *Saccharomyces cerevisiae trm7*Δ strain with Arabidopsis *SCS9* cDNA, and hypersensitivity of *scs9-2* seedlings to paramomycin and rose bengal. (**A**) Comparative growth curves of various *S*. *cerevisiae* strains grown in YPD at 30°C. Open squares represent wild-type strains (BMA64) transformed with plasmid p423-GAL1 alone (WT ccdB; broken red line) or using a plasmid carrying an Arabidopsis *SCS9* cDNA (WT SCS9; black line). Filled circles represent *trm7*Δ strain transformed with the plasmid alone (trm7 ccdB; dark circles) or with the plasmid carrying the Arabidopsis *SCS9* cDNA (trm7 SCS9; orange circles). (**B**) Col-0 and *scs9-2* seedling growth in MS plates alone or in the presence of 0.005% (w/w) and 0.01% (w/w) of paramomycin. (**C**) Quantitative analysis of paramomycin effects on growth retardation in Col-0 and *scs9-2* seedlings measured as reduction in fresh weight (FW). (**D**) Quantitative analysis of anthocyanins accumulation in Col-0 and *scs9-2* seedlings treated with paramomycin at the indicated concentrations. (**E**) Differential effects of rose bengal on growth inhibition of Col-0 and *scs9-2* seedlings grown in MS plates.

### *scs9* mutant is hypersensitive to paramomycin and rose bengal

The yeast *trm7*Δ strain has been described to be highly sensitive to paramomycin [13], an antibiotic of the aminoglycoside family that impairs translation by increasing codon misreading in prokaryotes and eukaryotes [29]. Therefore, we hypothesized if SCS9 and Trm7p are functional homologs, then a *scs9* Arabidopsis strain might also show enhanced sensitivity to paramomycin. The *scs9-1* strain carries the kanamycin resistance gene as a selectable marker, which might interfere with the antibiotic sensitivity assay; therefore we employed the *scs9-2* strain that instead carries resistance to the herbicide BASTA as the selectable marker. Col-0 seedlings were moderately sensitive to 0.005 to 0.01% paramomycin, which partially slowed plant growth and elicited moderate anthocyanin deposition in leaves, presumably as a consequence of antibiotic imposed stress (Fig 4B–4D). Interestingly, the *scs9-2* mutant showed enhanced sensitivity to the antibiotic, as indicated from the decreased seedling growth and a concurrent increase in anthocyanin deposition in leaves of paramomycin-treated *scs9-2* plants (Fig 4B–4D). These effects were more evident at 14 μM (0.01% w/v) compared to 7 μM (0.005% w/v) antibiotic concentration, which also maximized the differences between Col-0 and *scs9-2* seedling growth. Therefore, consistent with the yeast *trm7*Δ mutant, the Arabidopsis *scs9-2* mutant was also highly sensitive to paramomycin.

Moreover, Khoury *et al*. [30] reported the *trm7*Δ strain was more sensitive to oxidative stress and exhibited enhanced growth inhibition in the presence of reactive oxygen species (ROS) (i.e., H_2_O_2_). Therefore, we examined if the *scs9* mutant became similarly more sensitive to oxidative stress. We treated Arabidopsis seedlings with the synthetic dye rose bengal, which results in conditional ROS formation in the presence of light [31], and we compared the responsiveness of Col-0 and *scs9-2* seedlings to this agent. Col-0 seedlings grown in Petri dishes showed sensitivity after 5 days exposure to 2 μM rose bengal, which elicited partial chlorosis in leaves, reduction in root growth, and inhibition of lateral root formation (Fig 4E). *scs9-2* mutant seedlings exhibited increased sensitivity to the dye, which became bleached instead of chlorotic, and seedlings eventually died after 5 days exposure (Fig 4E). Therefore, both yeast *trm7*Δ and Arabidopsis *scs9* mutants displayed hypersensitive responses to this type of ROS-derived stress condition. In contrast, *scs9-1*, *scs9-2*, and Col-0 seedlings are equally sensitive to salt-derived stress as recorded in seedling growth inhibition and germination assays performed with increasing concentrations (i.e., 0, 50, 100, and 200 mM) of NaCl (S2 Fig). These differences might indicate a selectivity for this specific tRNA 2´-*O*-ribose methyltransferase in mediating adaptation to specific stressing situations.

### SCS9 localizes to the nuclei, including the nucleolus

tRNA molecules, although transcribed in the nucleus, function and are distributed in different subcellular compartments, emphasizing the importance of subcellular localization of tRNA modifying enzymes. Moreover, mature tRNA move in a retrograde direction from the cytoplasm to the nucleus via retrograde tRNA nuclear import, a process conserved from yeast to vertebrates, and proposed to function as a pathway that monitors end processing of pre-tRNAs and the modification state of mature tRNAs [32]. Our objective was to identify the cellular compartment where SCS9 exerted its function as a potential tRNAs modifier. We therefore used a SCS9 tagged to the fluorescent GFP or mCherry protein, which was functional in complementing the *scs9* phenotype (Fig 3E), and performed co-localization studies using confocal microscopy. The free GFP or specific subnuclear compartment marker proteins were used upon transient Agroinfiltration of *Nicotiana benthaminana* leaves with *Agrobacterium* strains carrying each corresponding gene construct. eIF4A, a RNA helicase component of the Exon Junction Complex (eiF4A-mRFP) and the histone H3 variant cenH3 (CENH3-mRFP) co-localized with SCS9-mCherry in the nucleolus and nucleoplasm (Fig 5; panels iv and v), indicating SCS9 partial enrichment or preference for the nucleolus. Coilin (Coilin-mRFP) and U2b´´(U2b´´-GFP), two Cajal Body markers and other nuclear bodies often associated with the nucleolus, also confirmed SCS9 localization in the nucleus, and its preference for the nucleolus but not for any type of nuclear bodies (Fig 5; panels ii and iii). Finally, free GFP, which accumulated in the cytoplasm and nucleus, but was excluded from the nucleolus, allowing a clear identification of SCS9-mCherry in the nucleolus (Fig 5; panel i). Therefore, we concluded that SCS9 is preferentially localized in the nucleus, and exhibited preference for the nucleolus. These results suggested modifications of tRNA molecules, directed by the methyltransferase enzyme, most likely occur in the nucleus and not the cytoplasm.

**Fig 5:** SCS9 nuclear localization. Co-localization patterns of SCS9, fused to either GFP or mCherry, with free GFP (panel i) and several different nuclear tagged proteins, including U2b” (panel ii), Coilin (panel iii), eIF4A (panel iv), and CENH3 (panel v) in epidermal cells from *N*. *benthamiana* transfected with each respective pair of constructs; evaluated by confocal microscopy.

### SCS9 is required for tRNA 2´-*O*-ribose methylation *in vivo*

Based on the close structural similarities between SCS9 and the *S*. *cerevisiae* Trm7p, *E*. *coli* FtsJ/RrmJ, and human FTSJ MTases, we tested whether SCS9 was similarly involved in 2´-*O*-ribose methylation of nucleotides in the Arabidopsis tRNAs anticodon loop. Positions 32 and 34 in the anticodon loop (Fig 6A) were identified as targets of Trm7p-like MTases [13]. In addition, when position 32 of a given tRNA was 2´-*O*-methylated, the wobble position 34 of the same tRNA was 2´-*O*-methylated by the same enzyme. Modified nucleotides corresponding to Arabidopsis tRNAs potentially altered due to defects in SCS9 were identified by comparing Col-0 modifications with those that commonly differed in *scs9-1* and *scs9-2* mutants. We used young seedlings as a source of plant material, which according to our previous experiences, show higher abundance of RNA. tRNA isolation, degradation, and subsequent HPLC analysis of separated nucleosides were performed as previously described [6]; elution time and spectrum of each peak were used to identify different modified nucleosides. Characteristic chromatograms of Col-0, *scs9-1* and *scs9-2* plants are shown in S2 Fig. Twenty-one major modified nucleosides were detected in the three genetic backgrounds, which all fit into previously identified modifications in Arabidopsis [6]. Notably, HPLC chromatogram comparison between Col-0 and the two mutants revealed *scs9-1* and *scs9-2* plants carried identical conspicuous diminutions in 2-*O*-methylated cytidine (Cm) content when compared to other invariant modified nucleosides such as 7-methyl guanosine (m^7^G) or 1-methyl guanosine (m^1^G) (S3 Fig). Cm modified nucleosides showed 70% reduction in *scs9-1* and *scs9-2* plants compared to Col-0 plants (Fig 6B). In addition, 2´-*O*-methylated uridine (Um) content showed a 30% reduction in both mutants (Fig 6B). However, in *scs9-1* and *scs9-2* mutants the decrease in 2-´*O*-methylated guanosine (Gm) was consistently much less, at only 10–15% reduction (Fig 6B). More accurate and straightforward determination of 2-*O*-methylated cytosine (Cm) content by LC-MS confirmed the notable reduction observed by HPLC analysis in *scs9-1* and *scs9-2* plants when compared to Col-0 plants (Fig 6C). Interestingly, following *P*.*s* DC3000 inoculation, Col-0 plants showed a moderate but progressive accumulation of Cm with a statistically significant 60% enhancement occurring at 72 and 120 h.p.i when compared to its control at 0 h.p.i. (Fig 6C). Conversely, *scs9-1* and *scs9-2* plants were impaired in this pathogen-mediated enhancement of Cm (Fig 6C). For Um nucleoside modification (Fig 6C), and to a lesser extent also for Gm (S4 Fig), LC-MS quantification revealed similar enhanced accumulation in Col-0 at 72–120 h.p.i. These enhancements were not observed to occur in *scs9-1* and *scs9-2* plants (Fig 6C and S4 Fig).

**Fig 6:** Reduced content of tRNA-derived 2’-*O*-methylcytosine (Cm), 2’-*O*-methyluracil (Um) and 2’-*O*-methylguanine (Gm) in *scs9-1* and *scs9-2* mutants. (**A**) Position of common modifications found in cytoplasmic tRNA in Arabidopsis and its major domains. tRNA is shown in its common secondary structure form, with circles representing nucleotides and lines representing base pairs. Position in shaded grey indicates the proposed tRNA methylation site for Trm7-like MTases in eukaryotes. Residue 34 corresponds to the wobble nucleotide. AAS (amino acid-accepting stem); DSL (dihydrouridine stem and loop); ASL (anticodon stem loop); VL (variable loop). Conventional abbreviations for nucleotide modifications are used; see the Modomics database (http://modomics.genesilico.pl). (**B**) Percent reduction of Cm, Um, and Gm content in *scs9-*1 and *scs9-2* relative to Col-0 plants as determined by HPLC analysis. Each value was relative to the amount of tRNA-derived 7 methylguanosine (m^7^G) and 1-methylguanosine (m^1^G), which remained invariant in all the genotypes. Data points represent the average of three biological replicates. (**C**) Relative content of Cm and Um modified nucleosides in Col-0, *scs9-1* and *scs9-2* plants during the course of an infection wit *P*.*s*. DC3000 as determined by LC-MS. Samples were taken at 0, 24, 48, 72 and 120 h.p.i. Each value was relative to the amount of tRNA-derived 1-methylguanosine (m^1^G) which remained invariant during the infection process. Data represent the mean ± SD; n = 3 replicates. Asterisks indicate statistical differences compared with its respective genotype as referred to its time 0 control (P<0.05) analyzed using a Student’s t-test. (**D**) tRNA Northern blot in mock- and *P*.*s*. DC3000-inoculated Col-0, *scs9-1*, and *scs9-2* plants. Leaf samples were collected at 3 d.p.i. The membranes were hybridized with radiolabel probes to tRNA^Phe^, tRNA^Gln^, tRNA^Leu^, tRNA^Trp^. Equal RNA loading was verified by staining with EtBr (low panel).

The three nucleoside modifications are highly conserved modifications in the tRNA anticodon loop, Cm occurring at positions 32 and 34, Um at position 32, and Gm at position 34 (Fig 6A). Positions 32 and 34 are known targets of Trm7p-like MTase, it is therefore likely that SCS9 is similarly required for 2´-*O*-ribose methylation at position 32 and 34. In yeast, Wilkinson *et al*. [33] reported cytosine and uracil nucleotides at position 4 of tRNAs (Fig 6A) were also 2-*O*-methylated; however at this position ribose methylation was Trm7p-independent, and instead required the Trm13p methyl-transferase. It remains unknown whether Um and Cm at position 4 occurs in plants, and if a Trm13-like enzyme regulates these specific modifications.

The 2´-*O*-ribose modifications at positions 32 and 34 of the anticodon loop revealed by our study occurred in tRNA^Phe(GmAA)^, tRNA^Trp(CmCA)^ and tRNA^Leu(UmAA)^ [3,13]. Reduced 2´-*O*-methylated nucleoside accumulation observed in *scs9-1* and *scs9-2* mutants might result from reduced accumulation of the respective tRNA precursors. We therefore performed Northern blots of small RNAs extracted from Col-0 and the two *scs9* mutants, and hybridized the filters with radiolabeled probes specific for each of the three indicated tRNAs. The non-related tRNA^Gln^ was used as an internal control. Noticeable changes in RNA accumulation were not observed in any genetic backgrounds for any tRNAs examined (Fig 6D). In addition, alterations in tRNA content were not detected following *P*.*s*. DC3000 inoculation.

Therefore, the marked reduction in Cm and Um accumulation, and to a minor extent in Gm, common to the *scs9* mutants, is a consequence of 2´-*O*-methyl transferase loss-of-function, and which appeared to have no effect on transcript levels of corresponding tRNAs.

### Other tRNA modifications are not essential for plant immunity

Modifications based on methylation (e.g., m^1^G, m^2^G, m^2^_2_G, m7G, m^5^U, m^5^C, m^1^A, m^1^I, Am, Cm, Um, Gm) were most common from the 21 different tRNA alterations detected in Arabidopsis and poplar [6]. Moreover, bioinformatic analysis of the Arabidopsis genome resulted in identification of 90 predicted homologous modification genes for modifications found in plants, except for genes responsible for m^2^A and m^6^A alterations which were not available, and the *TsaA* gene for m^6^t^6^A modification, which did not provide any homologous Arabidopsis gene [6]. Therefore, we questioned if the absence of another tRNA methyltransferase type could affect plant immunity to the same extent as the elicited by the absence of Trm7p-like SCS9 methyltransferase. Consequently, we identified various T-DNA insertion mutants interrupting the ORF for a selected group of homologous *TRM*-*like* genes encoding distinct tRNA modifying enzymes (Fig 7A). Results suggested none of the selected tRNA methyltransferase encoding genes from Arabidopsis were essential, and the phenotype of the mutant lines revealed no difference to the wild-type Col-0 in terms of growth and developmental habits, except for the *trm9*-*like* mutant which showed slight growth retardation (S5 Fig).

**Fig 7:** *trm-*like mutants and disease resistance to *P*.*s*. DC3000. (**A**) Diagram showing T-DNA insertions occurring in the indicated exons of genes encoding TRM-like methyltransferases from Arabidopsis: At3g02320 is homologous to TRM1; At2g22400 is homologous to TRM4; At3g56120 is homologous to TRM5; At1g36310 is homologous to TRM9; At5g47680 is homologous to TRM10; At5g14600 is homologous to TRM61. Exons are indicated with solid rectangles. T-DNA insertions are indicated with red rectangles. Distances are only approximate. (**B**) Growth rates of *P*.*s*. DC3000 in Col-0, *scs9-1*(*trm7-like*), *trm1-like*, *trm4-like*, *trm5-like*, *trm9-like*, *trm10-like*, and *trm61-like* plants. Shown is the bacterial growth measured at three days after inoculation in each of the indicated genotypes. Error bars represent standard deviation (n = 12). Asterisks indicate statistical differences to Col-0 (P<0.05) using Student’s t-test.

At3g02320 is one of three genes homologous to *TRM1*, which codes for a tRNA methyltransferase for dimethylguanosine modification (m^2^_2_G) at position 26 in *S*. *cerevisiae* [34] (S5 Fig). The yeast Trm4p protein catalyzes formation of m^5^C at positions 34, 40, 48, and 49 [35], and eight homologous genes belonging to the NOP1/NOP2/Sun protein family are present in Arabidopsis; we arbitrarily selected At2g22400 among these genes. At3g56120 is one of three Arabidopsis genes with homology to TRM5 from yeast encoding tRNA (m^1^I) methyltransferase, which cooperates with the deaminase Tad1p for deamination of A to I at positions 34 and 37 in the anticodon loop [36]. *TRM61* and *TRM6* are genes coding for the two subunits of tRNA(m^1^A58) methyltransferase on the initiator tRNA^Met^ in yeast [37]. One *TRM61* homolog exists in Arabidopsis, At5g14600. At1g36310 was homologous to the yeast *TRM9* gene coding for tRNA methyltransferase which catalyzed esterification of modified uridin nucleotides resulting in formation of 5-methylcarbonylmethyluridine (mcm^5^U) at the wobble position in tRNA^Arg,Glu^ [9]. Finally, At5g47680, represents the only homologue of the yeast *TRM10* gene, coding for a tRNA methyltransferase involved in modification of m^1^G at position nine of 10 different tRNA species [38]. We subsequently examined if these *trm*-*like* mutants were defective *P*.*s*. DC3000 immune response as in *scs9* mutants. Upon bacterial inoculation, none of the mutant strains seemed to be affected in the immune response, at least to the extent observed for the *scs9* mutant (Fig 7B). Only partial, but not statistically significant enhancement in bacterial growth compared to Col-0 was observed for the *trm10*-like mutant. The results therefore suggested a SCS9-mediated specific Cm and Um requirement at positions 32 and 34 of the anticodon loop of specific tRNAs for plant immunity towards *P*.*s*. DC3000. In any case, at this stage we cannot rule out that for some selected TRM-like methyltransferases, the existence of paralogous genes might mask the phenotype of single mutant strains, condition that nevertheless does not seem to apply in TRM7-like SCS9.

## Discussion

In the present study, we employed a variety of approaches to define a relationship between specific tRNA modifications at the anticodon loop, and the execution of an effective immune response towards *P*.*s*. DC3000 in Arabidopsis. The *scs9* mutant identification, which suppressed the previously described *csb3* mutant *P*.*s*. DC3000 resistant phenotype, indicated that SCS9 was pivotal for plant resistance towards this pathogen. In *scs9* plants the molecular hallmarks associated with activation of immune responses were properly activated; however, despite these measures *scs9* plants were unable to fend off *P*.*s*. DC3000. Therefore *scs9* plants posses a critical distinction that differentiates *scs9* from other mutant plants with a similar compromised immunity. NPR1 is the central regulator of SA-mediated plant immunity towards *P*.*s*. DC3000 [39], and therefore the *npr1* mutant is unable to resist *P*.*s*. DC3000. However, at variance with the *npr1* mutant, *scs9* plants are not compromised in SA perception and neither on its accumulation. This makes a clear distinction between *npr1* and *scs9* plants, suggesting that the defect(s) in *scs9* plant immunity control operate downstream or distant to the point of *npr1* failed control.

Map-based cloning revealed SCS9 is homologous to yeast Trm7p [13], human FTSJ1 protein [26], and bacterial FtsJ/RrmJ [25] proteins, encoding 2´-*O*-ribose tRNA methyltransferases. These enzymes exhibited the common “MTase fold” [28], suggesting their biological target tRNA must be similar. In fact, SCS9 provided the fission yeast Trm7p functions, demonstrated by effective complementation of a *trm7*Δ mutant using Arabidopsis *SCS9* cDNA, and providing unequivocal evidence the *SCS9* gene is the Arabidopsis functional homolog of the *TRM7* gene. The mechanistic relationship between Trm7p and SCS9 was further established by the observation that loss of either protein makes corresponding *trm7*Δ and *scs9* mutant cells sensitive to oxidative stress and also sensitive to paramomycin, an antibiotic that impairs translation by increasing codon misreading [29]. However, this enhanced sensitivity of the *scs9* mutants is not manifested when other type of abiotic stress, such as saline stress, is imposed. These results thus give support to the importance of this specific tRNA 2´-*O*-ribose methyltransferase for plants to selectively cope with only certain types of stress. Moreover, consistent with *trm7*Δ, Arabidopsis *scs9* plants were defective in the 2´-*O*-ribose methylation of nucleotides 32 and 34 of the tRNAs anticodon loop. The marked reduction in 2-*O*-methylated cytosine (Cm) content, not as notably reduced in Um and Gm at nucleotides 32 and 34, which are targets of yeast Trm7p MTase [13], reinforced our conclusion that Arabidopsis SCS9 and yeast Trm7p MTases are homologous. Furthermore, the observation that Cm content, and to a similar extent also Um content, enhance upon infection of Col-0 plants with *P*.*s*. DC3000, and that their deficiency correlates with a defective immune response, gives relevance to SCS9 as a new component regulating effectiveness of plant immune responses. Moreover, the lack of defects in *scs9* mutants in activating rapid immune responses suggests that the point of control of SCS9 is to regulate the final outcome of the immune response without interfering early stages of immune signaling. Our observation on the importance of tRNA modification in biotic stress response thus adds to the observation of Pajerowska-Mukhart *et al*. [40] who reported that the levels of uncharged tRNA corresponding to phenylalanine were shown to rapidly, and transitorily, increase in response to pathogen attack to allow translation of TBF1, a key defense regulator important to mediated SA-mediated immunity. Even though this latter study focused on a different regulatory step of translation in plant immunity, the evidences also points towards the importance of tRNA metabolism as a point of control regulating biotic stress adaptation.

How then, can a defect in 2-*O*-methylated cytosine (Cm) at specific tRNAs wobble positions interfere with plant immunity while maintaining an intact upstream signal transduction pathway normally required for mounting an efficient plant immune response? We speculated that following *P*.*s*. DC3000 inoculation, reprogramming of specific tRNAs wobble modifications led to selective translation of mRNA species enriched with the cognate codon, in a manner similar to that described in other eukaryotes [41,42]. The absence of accurate modifications at the wobble position in specific tRNAs would drive inefficient translation or generate misreading of specific proteins, which would be vital for an effective immune response. This translational control is congruent with SCS9 operating downstream of NPR1, and of its subordinated transcriptional reprograming, during the immune response. It is important to note that the derived phenotypic defects due to the absence of a correct tRNA 2-*O*-methylated modification were conditional, since *scs9* plants suffered no penalty in normal development, with only minor growth retardation. Moreover, *scs9* mutants carried no gross alterations at the protein synthesis and accumulation levels, as deduced from normal protein pattern observed in SDS polyacrylamide gels, or from the normal accumulation of host induced pathogenesis-related proteins (e.g., PR-1), interpreted from Western blot analysis. This favors a hypothesis where defects derived from *scs9* mutations would very likely elicit impacts at the proteome level in a very specific manner, presumably affecting only translation in a selective group of proteins with a pivotal role for effective execution of the immune response program. The literature provides some evidence for specific tRNA modification-dependent translation control during stress response in higher eukaryotes, and particularly to oxidative stress. For example, Kalhor and Clarke [9] showed yeast Trm9 catalyzed methyl esterification that led to conversion of uracil into mcm^5^U at the wobble position of tRNA^Arg(UCU)^ and tRNA^Glu(UUC)^. This process enhanced binding of the anticodon, and therefore, facilitated translation of AGA- and GAA-rich transcripts, which functionally maps to processes of stress signaling to fend off deleterious effects of ionic radiation on DNA damage [43]. Similarly, Trm4, which catalyzes m^5^C at the wobble position of tRNA^Leu(CAA)^ enhanced translation efficiency of mRNAs enriched in the UUG codon recognized by this tRNA, and loss of Trm4 caused hypersensitivity to the cytotoxic effects of H_2_O_2_ [38]. One of these UUG-biased mRNAs whose translation is controlled by Trm4 is the ribosomal protein Rpl22A, whose increase in translation is required to cope with oxidative stress [44]. This observation adds to a growing recognition of the role for functional diversity in ribosome composition and for ribosomes in selective translation of proteins [45]. Interestingly, this reprograming of the translation machinery reconciles with the proposed generation of “immunoribosomes” as a subset of T-cell ribosomes, responsible for translating peptides involved in antigen presentation [46]. These are only examples illustrating towards the enormous complexity underlying translation control mechanisms, and our limited understanding, particularly in plants. Therefore, the variety of tRNA modifications, its complex regulation, and the established biases in gene codon distributions, points towards the existence of mechanisms evolved to fine tune the translational response to any cell stimulus; as those suggested to regulate immunity by SCS9.

Our results also led to hypothesized that the absence of specific methylation at the wobble position of the selective group of tRNAs controlled by SCS9 might affect the synthesis of a codon-biased cognate protein(s) required for passive resistance to the pathogen, which might function as a repressor protein(s). If the repressor is defective or poorly translated, then a cellular factor or molecular process might become de-repressed, which in turn might favor bacterial growth and host colonization. This latter explanation is also congruent with SCS9 controlling a non-immunity related plant process that might regulate plant susceptibility to pathogens by operating at different levels, from pathogen attraction and attachment to the host to nutrient production and transport from the host, as described in several studies [47]. This may reconcile with the existence of tRNA cleaving toxins, developed by certain microbes to act on specific positions within the anticodon loop of target tRNAs, such as colicin and onconase [4], or the γ-toxin of *Kluyveromyces lactis* that targets and cleaves specific tRNAs in the yeast *S*. *cerevisiae* that have the mcm^5^s^2^U modification at position 34 of tRNA^Glu(UUU)^ [48]. At this stage we can not disregard that bacterial effector proteins may have been developed to target specific modified plant tRNAs, or even the MTase responsible for such tRNA modification, as part of a pathogenic strategy.

We cannot ignore the possibility of a surveillance mechanism leading to hypomodified tRNAs degradation as part of a conserved response to stress [49,50], which might have a potential impact on translation and disease progression, as described by Thompson and Parker [11]. The emergence of tRNA-derived fragments (tFRs) as a novel class of small regulatory RNAs [51,52] with potential roles as regulators of gene silencing [53,54], and as part of a conserved stress response also described in plants [55], might therefore interfere with epigenetic processes governed by small RNAs, such as RNA-directed DNA methylation (RdDM), which has recently been demonstrated as pivotal for plant immunity to *P*.*s*. DC3000 [56]. However, this later mechanism seems less likely, since the hypomodified tRNAs levels in *scs9* plants appeared not to be degraded, not even following inoculation with the pathogen.

In summary, the present results denote the importance of keeping intact tRNA modifications for mounting an effective immune response. Unraveling further components, its regulation and identifying target proteins whose translation is regulated by these tRNAs modifications will open new avenues to better understand how the effectiveness of immune responses is regulated in plants.

## Methods

### Plants growth conditions

*Arabidopsis thaliana* plants were grown in a growth chamber (19–23°C) on a 10-hr-light and 14-hr-dark cycle as previously described [23]. All mutants are in Col-0 background.

### GUS staining and callose deposition analysis

Plant leaves were incubated overnight at 37°C in GUS staining buffer as previously described [57]. For callose deposition analyses, leaves were stained with aniline blue and callose deposition quantifications were performed as described by Garcia-Andrade *et al*. [57].

### Mapping and cloning

The *scs9* mutant was backcrossed twice to the *csb3* line to confirm its recessive inheritance. *scs9* plants were crossed to L*er*, and F1 plants were allowed to self. F2 plants were scored for co-segregation of enhanced disease susceptibility to *P*.*s*. DC3000 with simple sequence length polymorphisms (SSLP) [56,58]. Molecular markers were derived from the polymorphism database between the L*er* and Col-0 ecotypes (http://www.arabidopsis.org). Whole genome sequencing and identification of nucleotide polymorphisms was carried out at the John Innes Centre (Norwhich, UK) as a genome service exchange using an Illumina GAIIx platform and the bioinformatic pipeline devised by Austin *et al*. [24]

### Gene constructs, expression in yeast and transgenic plants

To amplify *SCS9* cDNA, PCR was performed using the Expand high-fidelity PCR system (Roche) with 1 μL of cDNA using BPSCS9Fw and BPSCS9Rv specific primers including Gateway adapters and recombined to pDONR221 using Gateway technology (Life Technologies) and recombined into the different destination vectors using LR ClonaseMixII kit (Invitrogen). List of primers used for cloning purposes is provided in Supplementary information. For the *SCS9-GFP* overexpressing construct, pDONR221 SCS9 was recombined to pB7FWG destination. For the SCS9-mCherry overexpressing construct, pDONR221 SCS9 was recombined to the modified pEarlyGate101 vector [57]. For the yeast *trm7* complementation assay, pDONR221 SCS9 vector was recombined to the yeast expression vectors p423-GAL1 and p432-GAL1-GFP to generate p423 GAL1/SCS9 and p423 GAL1/SCS9-GFP respectively. Sequencing of individual clones confirmed that there were no errors in the *SCS9* cDNA. p423 GAL1/SCS9, p423 GAL1/SCS9-GFP and the respective empty vectors were transformed into wild-type (BMA64, MATα; [13]) and trm7p (YBL4409, MATα, trm7Δ:TRP1 [13]) yeast strains as previously described [59] and grown on minimal medium agar plates lacking His. Individual yeast transformants were then transferred to selective liquid media containing 2% (w/v) Gal to induce expression of *SCS9*. These cultures were incubated at 28°C for 2 d and then were adjusted to OD600 = 0.1 to perform the time-course growing assays.

### Transient expression in *Nicotiana benthamiana* leaves

Almost fully expanded leaves were infiltrated with a suspension of *Agrobacterium tumefaciens* C58 bearing the relevant construct in 10 mM MES pH 5.6, 10 mM MgCl2, 150 mM acetosyringone at an OD600 = 0.5. After 2–3 days, fluorescence was analyzed in infiltrated leaves by confocal microscopy. For co-infiltration, Agrobacterium cultures grown separately and processed as indicated above, were adjusted to an OD600 = 0.5, and mixed prior to infiltration. Agrobacterium expressing the viral silencing suppressor P19 was included in all infiltrations.

### Confocal laser-scanning microscopy

Plant tissue was observed with a Leica TCS LS spectral confocal microscope using and HCX PL APO 640/1.25–0.75 oil CS objective. GFP-derived fluorescence was monitored by excitation with 488- and 514-nm argon laser lines, respectively, and emission was visualized with a 30-nm-width band-pass window centered at 515 nm. When RFP and mCherry were used, excitation was performed by means of a 543-nm green-neon laser line, and fluorescence emission was collected at 695 to 630 nm.

### RT-qPCR

Total RNA was extracted using TRIzol reagent (Invitrogen) following the manufacturer’s recommendations and further purified by lithium chloride precipitation. For reverse transcription, the RevertAid H Minus First Strand cDNA Synthesis Kit (Fermentas Life Sciences) was used. Quantitative PCR (qPCR) amplifications and measurements were performed using an ABI PRISM 7000 sequence detection system, and SYBR-Green (Perkin-Elmer Applied Biosystems). *ACTIN2* was chosen as the reference gene. Primers for amplicons covering each of the genes studied are listed below in Supplementary information.

### Western blots

Protein crude extracts were prepared by homogenizing frozen leaf material with Tris-buffered saline (TBS) supplemented with 5 mM DTT and protease inhibitor cocktail (Sigma-Aldrich). Protein concentration was measured using Bradford reagent; unless otherwise indicated 20 μg of total protein was separated by SDS-PAGE (12% acrylamide w/v) and transferred to nitrocellulose filters. The filter was stained with Ponceau-S after transfer, and used as a loading control. Immunoblots were incubated with the indicated primary antibodies at the appropriate dilution and developed by chemiluminescence using an anti-IgG peroxidase antibody (Roche) at a 1:1000 dilution and Western Lighting plus-ECL substrate (Perkin-Elmer).

### *Pseudomonas syringae* DC3000 inoculations

Arabidopsis leaves were infiltrated with *P*.*s*. DC3000 as previously described [23].

### T-DNA Arabidopsis mutants

T-DNA insertion mutants and primers used to identify insertions by PCR are listed in Supplementary information.

### tRNA isolation, digestion, HPLC and LC-MS analysis

Total RNA was extracted using Trizol Reagent (Invitrogen), small RNAs were separated from rRNA and mRNA using LiCl and tRNA was further purified using cellulose DE52 resin (Whatman Cat.#4057–200) as described in [6]. 100 μg tRNA dissolved in MQ water was degraded to nucleosides with P1 nuclease (Sigma Aldrich Cat.#54576-84-0) and alkaline phosphatase (TOYOBO, Japan Cat.#CAP-101) as described [6]. The modified nucleosides were analyzed using Reverse-phase HPLC (Waters Alliance HPLC system and Waters Absorbance Detector 2996) and a C-30 column (Develosil C-30 reverse-phase column, 250 × 4.6 mm; Nomura Chemical Co., Ltd.). The buffer gradient was as described [6]. Modified nucleosides were quantified relative to two internal standards (m^7^G and m^1^G). For LC-MS analysis, total RNA and microRNA was extracted using a microRNA extraction kit (Omega Bio-tek Inc.). RNA concentration was determined using NanoDrop ND-1000 spectrophotometer (Thermo Scientific), about 20ug tRNA was digested with 2U P1 nuclease (Sigma, N8630) and 1.5unit of Calf-Intestine Alkaline Phosphatase (TOYOBO, CAP-101) in 20ul of 20mM HEPES-KOH(pH7.0) at 37°C for 3 hours. Sample was diluted with MilliQ water (Millipore SYNNERGY) to a concentration of 5ug/ml, the injected volume was 10ul. API 4000 Q-TRAP mass spectrometer (Applied Biosystems) was used with an LC-20A HPLC system and a diode array UV detector (190−400 nm) equipped with an electro spray ionization source. ESI-MS was conducted in a positive ion mode. The nebulizer gas, auxiliary gas, curtain gas, turbo gas temperature, entrance potential, and ion spray voltage were 60 psi, 65 psi, 15 psi, 550°C, 10 and 5500 V respectively. Multiple reaction monitoring (MRM) mode was performed to determine parent-to-product ion transitions. Inertsil ODS-3(2.1 mm × 150 mm, 5 um particle size; Shimadzu) reversed-phase column with an Inertsil ODS guard column (4 mm x 10 mm, 5 μm particle size; Shimadzu) was used for chromatographic separation of nucleosides. The mobile phase gradient consisted of 2 mM ammonium acetate (solvent A) and methanol (solvent B). The flow rate was 0.6 ml/min at ambient temperature. Nucleoside standard uridine, cytidine, adenosine, guanosine, 1-methyladenosine, 7-methylguanosine, 5-methyluridine and 2’-O-methylguanosine nucleoside standards (Santa Cruz Biotechnology) were used to distinguish nucleoside isomers. The relative abundance of each selected modified nucleoside was calculated as area of the peak with the correct mass and parent-to-product ion transition, divided by total area for uridine, cytidine, adenosine and guanosine monitored nucleosides.

### Anthocyanin and SA quantification

Anthocyanin extraction and quantification was performed as previously described [60]. SA extraction and quantification was performed as described [61,62].

### Paramomycin and Rose Bengal assays

Seeds were sterilized and plated on MS medium (Duchefa Biochemie) supplemented with 0.5% sucrose, then stratified in darkness at 4°C for 3 days and transferred to growth chambers. To conduct paromomycin rate assay, seeds were plated on MS medium without or with paromomycin. The pictures were taken after 14 days. To conduct Rose Bengal assay, seeds sown on MS plates were stratified for 3 days at 4°C and were vertically grown for 4 days under normal conditions, and then seedlings were transferred to vertical square MS plates with or without 2 μM Rose Bengal. The pictures were taken after 7 days.

### tRNA blot analysis

20 μg of total RNA was electrophoresed on 2.5% agarose gels containing formaldehyde and blotted onto Nytran membranes (Schleicher & Schuell, Dassel, Germany) as described [60]. Equal loading of RNA was verified by ethidium bromide staining of the gel before transfer to the membrane. Oligonucleotide probes were ^32^P-labeled with T4 polynucleotide kinase (Fermentas) according to manufacturer’s instructions and then purified on a microspin G-25 column separating labeled probe from unincorporated nucleotides. Hybridization and washing conditions of filters were as described [63].

### Flg22 treatments and NaCl growth assay

For flg22 treatment seedlings were grown and treated with 1 μM flg22 as previously described [64]. For saline growth assay and effect on germination, sterilized seeds were plated on MS solid supplemented with 0.5% sacarose and MES (0.01%), and without or with NaCl (at different concentrations). Pictures and data of fresh weight were taken after 13 days. To analyze the seedling growth inhibition by salt stress, seeds sown and grown under normal conditions (without NaCl) for 6 days, were transferred to MS medium without and with NaCl (at different concentrations). Pictures and data of fresh weight were taken after 7 days of treatment. 20 seedlings were analyzed for each replicate.

## Supporting Information

S1 Fig Arabidopsis SCS9 amino acid sequence alignment with tRNA MTases from *S*. *cerevisiae* (Trm7p), *H*. *sapiens* (FTSJ1), and *E*. *coli* (FtsJ/RrmJ). Identical and chemically equivalent residues are indicated with black asterisks and dots, respectively. Conserved motifs have been labeled according to the nomenclature proposed by Pósfai *et al*. [27], and are shown in blue. Predicted interactions with AdoMet and the methylated nucleotide of tRNA are designated by blue dots and red triangles, respectively. The predicted catalytic tetrad K-D-K-E is labeled with red asterisks and red shading. The blue arrow denotes the amino acid residue mutated in the *scs9* mutant.
(TIF)

S2 Fig Seed germination (A) and seedling growth (B) inhibition assays by NaCl. Quantitative analysis of effect on germination of seeds (A) and growth inhibition (B) of Col-0, *scs9-1* and *scs9-2* seedlings following application of different NaCl concentrations (0, 50, 100 and 200 mM), measured as reduction in fresh weight (%). Data represent mean ± SD; n = 3 replicates. A representative MS plate of each condition with three genotypes is shown.
(TIF)

S3 Fig HPLC chromatogram of modified tRNA-derived nucleosides. tRNA purified from plant tissue was digested with P1 nuclease and treated with alkaline phosphatase. The modified nucleosides were analyzed using Reverse-phase HPLC and a C-30 column. The chromatogram shows nucleoside peaks derived from Col-0 (A, D), *scs9-1* (B, E) and *scs9-2* (C, F) plants. X-scale: retention time in minutes. Y-scale: UV absorbance at 254nm. Four major peaks and m^7^G (7-methylguanosine) are marked with lines which served as chromatograms references. Cm (2’-O-methylcytosine), Um (2’-*O*-methyluracil), and Gm (2’-*O*-methylguanine) peaks are marked with arrows.
(TIF)

S4 Fig Effect of *P*.*s*. DC3000 on Gm nucleoside content in Col-0, *scs9-1* and *scs9-2* seedlings. Relative content of Gm nucleosides in Col-0, *scs9-1* and *scs9-2* seedlings after a *P*.*s*. DC3000 infection was determined by LC-MS. Samples were taken at 0, 24, 48, 72 and 120 h.p.i. Each value was relative to the amount of tRNA-derived 1-methylguanosine (m^1^G). Asterisks indicate statistical differences compared with its respective genotype as referred to its time 0 control (P<0.05) analyzed using a Student’s t-test.
(TIF)

S5 Fig Arabidopsis *trm* mutant phenotypes. (**A**) Normal development of different *trm*-like T-DNA insertion mutants observed at 35 days after sowing and grown in pots in the greenhouse. Note the absence of gross developmental defects except for *trm9*-like mutant whose growth was reduced. (B) Modified nucleosides in eukaryotic tRNAs. Clover-leaf structure of eukaryotic tRNA. Each circle represents a nucleoside, numbered from 5´-to-3´end. Modified nucleosides found at different positions are shown in bold. Arrows indicate the specific modification and nucleoside position in tRNA for each of the corresponding homologous TRM-like enzymes considered in the present study.
(TIF)

S1 Table Accumulation of PR-1 protein at different time points following *P*.*s*. DC3000 inoculation in Col-0, *scs9* and *npr1* plants (left table), and also following SA application in Col-0 and *scs9* plants (right table). Western blot bands, of the type shown in Fig 2H and 2I, were quantified using the ImageJ software. Band intensities of triplicate technical repeats of two biological independent experiments were quantified and relative levels to the corresponding Col-0 controls are presented as a percentage ± SD.
(TIF)

S1 Text Primer sequences. (DOC)
